The article "Cardiac Contractility Modulation Attenuates Chronic Heart Failure in a Rabbit Model via the PI3K/AKT Pathway" was retracted in 2024. Reasons: suspected computer-generated content; unreliable results or conclusions; concerns about the data; concerns about the results or conclusions.

# Cardiac Contractility Modulation Attenuates Chronic Heart Failure in a Rabbit Model via the PI3K/AKT Pathway

**DOI:** 10.1155/2020/1625362

**Published:** 2020-01-07

**Authors:** Qingqing Hao, Feifei Zhang, Yudan Wang, Yingxiao Li, Xiaoyong Qi

**Affiliations:** ^1^School of Graduate, Hebei Medical University, Shijiazhuang, China; ^2^Department of Cardiology Center, Hebei General Hospital, Shijiazhuang, China

## Abstract

The Akt plays an important role in regulating cardiac growth, myocardial angiogenesis, and cell death in cardiac myocytes. However, there are few studies to focus on the responses of the Akt pathway to cardiac contractility modulation (CCM) in a chronic heart failure (HF) model. In this study, the effects of CCM on the treatment of HF in a rabbit model were investigated. Thirty six-month-old rabbits were randomly separated into control, HF, and CCM groups. The rabbits in HF and CCM groups were pressure uploaded, which can cause an aortic constriction. Then, CCM was gradually injected to the myocardium of rabbits in the CCM group, and this process lasted for four weeks with six hours per day. Rabbit body weight, heart weight, and heart beating rates were recorded during the experiment. To assess the CCM impacts, rabbit myocardial histology was examined as well. Additionally, western blot analysis was employed to measure the protein levels of Akt, FOXO3, Beclin, Pi3k, mTOR, GSK-3*β*, and TORC2 in the myocardial histology of rabbits. Results showed that the body and heart weight of rabbits decreased significantly after suffering HF when compared with those in the control group. However, they gradually recovered after CCM application. The CCM significantly decreased collagen volume fraction in myocardial histology of HF rabbits, indicating that CCM therapy attenuated myocardial fibrosis and collagen deposition. The levels of Akt, FOXO3, Beclin, mTOR, GSK-3*β*, and TORC2 were significantly downregulated, but Pi3k concentration was greatly upregulated after CCM utilization. Based on these findings, it was concluded that CCM could elicit positive effects on HF therapy, which was potentially due to the variation in the Pi3k/Akt signaling pathway.

## 1. Introduction

Chronic heart failure (CHF) is the terminal stage of various structural and functional cardiac diseases [1]. This disease can cause a progressive reduction in cardiac output since it depresses the cardiac contractility and influences the conduction pathways as well by causing a delay in the onset of right or left ventricular systole [2,3]. Although many efforts have already been attempted to treat the CHF in the past decades, such as beta-blockers of metoprolol, bisoprolol, bucindolol, nebivolol, atenolol, and carvedilol [4,5], it still is one of the most common and a complex disease to tackle, and as a result, approximately 30 percent of patients are suffering from this disease worldwide [6].

It is well known that the pathological cardiac dysfunction is contributed to myocardial hypertrophy and cell apoptosis [7], which is influenced by the Akt, a serine/threonine protein kinase, also known as protein kinase B [8]. The Akt is the effector of Pi3k and is essential during postnatal cardiac development that is achieved predominantly by hypertrophy rather than hyperplasia of individual cardiomyocytes [9]. It suggested that increasing Akt expression in cells could promote their hypertrophy and hyperplasia. The Akt also plays an important role in T-lymphocytes and prostate cells to promote lymphoma and prostate cancer [10]. Therefore, it is critical to investigate the variation in protein levels in a CHF model and then develop potential methods to prevent this disease from becoming worse.

Cardiac contractility modulation (CCM) is a series of nonexcitatory signals which can be applied during the absolute refractory period to enhance the strength of left ventricular contraction without increasing myocardial oxygen consumption [11,12]. The process of contraction force increasing is mediated by reversing the molecular remodeling and restoring the expression of several calcium-handling proteins in myocardial hypertrophy with heart failure (HF) [13]. Also, it was reported that CCM could significantly alter the cytoskeleton proteins and matrix metalloproteinases [14]. The Pi3k/Akt signaling pathway was activated by a serious of internal- and external-cellular proteins via the phosphorylation at Thr 308 and Ser 473 [8]. Therefore, the effects of CCM on attenuating the CHF are possibly contributed to the variation in Akt pathway signals and related proteins. Until now, there are few studies to focus on the responses of the Akt pathway proteins to the CCM in a rabbit model with HF. In this study, the effects of CCM application in rabbits with HF on their body and heart weight, heart beating rate, collagen volume fraction, Akt, FOXO3, Beclin, pi3k, mTOR, GSK-3*β*, and TORC2 expression in cardiac myocytes were investigated.

## 2. Materials and Methods

### 2.1. Animals

Thirty six-month-old healthy New Zealand white rabbits (2.5–3.5 kg) were obtained from the Experimental Animal Center of Hebei Medical University (HMU) and housed with 12-hour dark/light cycle for free access to food. This study complied with standards for the Care and Use of Experimental Animals of HMU and the Guide for the Care and Use of Laboratory Animals published by the US National Institutes of Health. All experimental procedures were approved by the Ethics Review of Lab Animal Use Application of Hebei Medical University.

### 2.2. Experimental Design and Management

The rabbits were randomly separated into three groups, namely, control, HF, and CCM groups, and each group contained 10 rabbits. The rabbits in the control group only received thoracotomy. The HF is characterized by the transition from an initial compensatory response to decompensation, which can be partially mimicked by transverse aortic constriction in rodent models [15]. Therefore, in the HF group, rabbits were treated by thoracotomy and ascending aortic cerclage. The rabbits in the CCM group suffered from thoracotomy, ascending aortic cerclage, and CCM application with a period of 4 weeks after HF occurred.

The rabbits in HF and CCM groups were anesthetized via the ear vein with 3% sodium pentobarbital at 1 ml/kg body weight, and their thoracic cavities were opened. Subsequently, their ascending aorta was dissected until the aorta circumference was constricted up to 60%. After 12 weeks, symptoms of heart failure occurred in the rabbits, including appetite reduction, breathing acceleration, and fewer activities. The HF model was thought to be successfully established while the left ventricular ejection fraction reached 40%.

Before the experiment, an electrode was used to deliver CCM. Specifically, one end of the electrode was sutured to the left ventricular anterior wall of rabbits, and the other end was punctured subcutaneously to the neck. Then, a cardiac stimulator (EPS320, BARD Micro-Pace, Inc., USA) was used to deliver CCM signals to the heart by sensed R-wave at the absolute refractory period. These signals consisted of biphasic square-wave pulses with phase duration of 2 ms, stimulus amplitude of 7 V, and 30 ms delay after R-wave sensing [16]. The CCM signals lasted 6 hours per day for a consecutive 4 weeks.

### 2.3. Sample Collection and Analysis

#### 2.3.1. Histology and Immunohistochemistry

At the end of the experiment, all rabbits were anesthetized with 0.5 mg/g tribromoethanol. Then, the hearts were fixed in 4% paraformaldehyde solution before storage for 10 min at −20°C. The hearts were sectioned transversely across myocardial papillary muscle before completely covered by paraffin. Myocardial histologic sections (5 *μ*m thickness) were slightly cut from the paraffin blocks and stained with 1% hematoxylin and eosin (H&E) and Masson's trichrome for 10 min at 37°C for histopathological analysis of myocardial fibrosis [17]. Afterward, all slices were fixed with 4% paraformaldehyde and photographed with a high-resolution digital microscope (×400; BX-51; Olympus, Tokyo, Japan). The collagen volume fraction (CVF) was calculated as the connective tissue areas divided by the total area of connective tissue and muscle [17].

#### 2.3.2. Western Blot Analysis

The total protein was obtained from leaf ventricular myocardial tissues after extraction with the RIPA lysis buffer (P0013B, Beyotime, Chine). Protein concentration was measured by the Pierce™ BCA Protein Assay Kit (Thermo Scientific, USA). A total of 60 *μ*g total protein was electrophoresed and separated with 10% SDS-PAGE and transferred onto nitrocellulose membranes (Millipore, US). After blocking with 5% fat-free milk at room temperature for 2 h, the membrane was incubated overnight at 4°C with primary antibody raised in mice against Akt (1 : 1000), FOXO3 (1 : 1000), Beclin (1 : 1000), Actin (1 : 1000), pi3k (1 : 1000), mTOR (1 : 1000), p-Akt (Ser473, 1 : 1000), GSK-3*β* (1 : 1000), and TORC2 (1 : 1000). All antibodies were purchased from Cell Signaling Technology (USA). Then, the membranes were incubated with HRP-conjugated secondary antibodies (1 : 2000; Cell Signaling Technology, USA) at room temperature for two hours. The immunoreactive bands were visualized using the enhanced chemiluminescence kit (ECL Millipore Corp., Bedford, MA, USA) in a western blotting detection system (Bio-Rad, CA, USA). Developed films were scanned and Image-ProPlus 5.1 was used for quantitative analysis. In this experiment, *β*-actin (1 : 1500, Bioss, Beijing, China) was used as the standard and the results were expressed as density values normalized to *β*-actin.

#### 2.3.3. Statistical Analysis

Data were presented as mean ± standard deviation. The main effect of treatment was analyzed by using Mixed proc in the SAS software (SAS 9.4 version, SAS institute, USA), and the differences among groups were analyzed using the LSD test. For the heart rate, the sampling dates were treated as a repeated measurement. Shapiro–Wilk was used to test the normality assumption on the residuals of each model, while residual plots were used to verify the homogeneity of variances. When the normality assumption was not met, response variables were transformed using the Box-Cox transformation. All analyses were performed using the Mixed procedure of SAS (SAS software, version 9.4, Cary, NC. USA) at a significant level of *p* < 0.05.

## 3. Results

### 3.1. Rabbits Survival and Healthy Conditions

At the end of this experiment, 27 rabbits survived (i.e., 9 rabbits in each experimental group), which met the criteria of HF. Their weight, including body and heart weight, significantly decreased for HF rabbits when compared with those in the control group and they progressively increased after CCM application (Table 1). The CCM signals significantly decreased the heart rate of HF rabbits, and similar heart beat rates were observed between rabbits in control and CCM groups (Table 1).

### 3.2. Effects of CCM Utilization on Histological Changes

Regarding the heart tissue section photomicrographs of different treatments stained with H&E, we observed the slightly disordered arrangement of myocardial cells, partial myocardial necrosis, and fibrous tissue proliferation and inflammatory cells infiltration in the HF group while compared with those in the control group. These pathological variations were partly recovered after the CCM application (Figure 1(a)).

To assess the changes in cardiac interstitial fibrosis, histological sections of the heart were stained with Masson's trichrome, and the CVF were also examined. Heart tissue in the HF group rabbits presented a massive and intensive collagen accumulation when compared with those in the control group (Figure 1(b)). But, the fibrotic heart tissue area greatly decreased after CCM application. Similar results were observed for the CVF, which indicated that it significantly increased after obtaining HF and then decreased obviously after CCM signals were applied (Figure 1(c)).

### 3.3. Effect of CCM on Heart Tissue Protein Expressions

In this study, three isoforms of Akt, including Akt1, Akt2, and Akt3, were investigated and they showed similar tendency after CCM application (Figure 2). Results of western blot analysis showed that CCM application and HF disease significantly increased the Akt levels, which suggested that HF and CCM upregulated Akt expressions in the rabbit model (Figure 2).

Compared with the control group, the expressions of FOXO3 and Beclin increased more significantly in the HF group and their concentrations markedly decreased after CCM treatment (Figures 3(a), 3(b), and 3(e)). Contrarily, Pi3k concentrations greatly decreased in rabbits of the HF group as compared with the control group, and it was significantly upregulated while the CCM signals were used to the HF rabbits (Figures 3(c)–3(e)). Compared with the control group, the mTOR, GSK-3*β*, and TORC2 expressions were sharply upregulated in the HF group and then significantly downregulated after CCM was used (Figure 4).

## 4. Discussion

The Akt family of serine-threonine kinases participates in diverse cellular processes, including the promotion of cell survival, glucose metabolism, and cellular protein synthesis in cardiac myocytes [8]. Generally, Akt contains three isoforms of Akt1, Akt2, and Akt3. In the heart, short-term Akt1 activation promotes cardiac growth [18], whereas long-term Akt1 activation induces pathological hypertrophy [19] because overexpression of the myristoylated form of Akt1 gene induces hypertrophy, leading to heart failure [20]. Similar to Akt1, Akt3 overexpression in the heart results in progression from adaptive to maladaptive hypertrophy [21]. In the rabbit model of our study, CCM operation significantly decreased the Akt1 and Akt3 levels, which are significantly lower than those in the HF group and higher than those in the control group (Figures 2(a) and 2(c)). Additionally, our results were supported by [22] reporting that Akt2 overexpression enhanced the murine sensitivity to cardiomyocyte apoptosis in response to ischemic injury. In our results, CCM application slightly decreased the Akt2 expression when compared with the HF group (Figure 2(b)), which could be potentially beneficial for the rabbits to partly recover from HF.

FOXOs are key transcription factors involved in multiple aspects of cardiac diseases. Generally, mammalian cells contain four FOXO isoforms of FOXO1, FOXO3, FOXO4, and FOXO6, and FOXO3 is the most abundant isoform expressed in hearts [23] and its metabolism in tissues was closely related to the Akt because Akt could control FOXO3 expression in the heart [24]. Thus, cardiac regeneration may be promoted by proper control of FOXO3 activity. Overexpression of Beclin, a proautophagy protein, stimulates autophagy and exacerbates cardiac dysfunction and pathological remodeling [25]. In our study, higher FOXO3 and Beclin expressions were observed in rabbits with HF compared with those in the control group, and CCM signals application significantly decreased their expressions (Figure 3). Wu et al. [26] reported that the activation of Pi3k expressions in the mouse heart could prevent cardiac remodeling. In this study, lower Pi3k expressions were observed in the HF group than in the control group, and their concentrations significantly increased in the CCM group (Figures 3(c) and 3(d)). Combining the results of FOXOs mainly plays a detrimental role [24], and Beclin expression causes the heart dysfunction; it was concluded that CCM is a potential method to attenuate HF by adjusting FOXO3, beclin, and Pi3k expressions in cardiac cardiomyocytes.

As reported from the previous literature, the anabolic effects of Akt are mediated, in part, through activation of mammalian target of rapamycin (mTOR) [27] and inhibition of glycogen synthase kinase-3*β* (GSK-3*β*). Activation of mTOR stimulates protein translation through its effects on p70 ribosomal S6 kinase (p70 S6K) and eukaryotic translation initiation factor 4E binding protein-1 (eIF4E-BP) [28]. However, Akt-mediated phosphorylation of GSK-3*β* [29] stimulates protein translation [30] by diminishing its inhibitory phosphorylation of eIF2B [31]. AKT (Ser473) is the downstream effector of mTORC2 [32], which means that while AKT (Ser473) is activated, suggesting that CCM could activate mTORC2 signaling. In the present study, we observed that CCM application significantly decreased the mTOR, GSK-3*β*, and TORC2 expression in myocardial cells in rabbits while compared with those in the HF group (Figure 4). Based on these findings, it was concluded that CCM therapy could prevent myocardial fibrosis in heart failure which is possibly related to the change in the PI3K/AKT signaling pathway in a rabbit model.

## Figures and Tables

**Figure 1:** Effects of cardiac contractility modulation (CCM) on myocardial histological changes (a) and (b) microphotography (400x) of myocardial samples from experimental rabbits. (c) Collagen volume fraction of rabbit myocardial tissues with different treatments. HF, heart failure. Different letters above each boxplot showed the significant differences at *p* < 0.05.

**Figure 2:** Effects of cardiac contractility modulation (CCM) on Akt1, Akt2, and Akt3 expression in different rabbit myocardial tissues under different treatments. (a) Akt1 expression; (b) Akt2 expression; (c) Akt3 expression; and (d) western blot images of Akt1, Akt2, and Akt3. CK, control group; HF, heart failure. Different lower letters above each boxplot showed the significant differences at *p* < 0.05.

**Figure 3:** Effects of cardiac contractility modulation (CCM) on FOXO3, Beclin, Pi3k(*α*110), and Pi3k(*α*85) expression in different rabbit myocardial tissues under different treatments. (a) FOXO3 expression; (b) Beclin expression; (c) Pi3k(*α*110) expression; (d) Pi3k(*α*85) expression; and (e) western blot images of FOXO3, Beclin, Pi3k(*α*110), and Pi3k(*α*85). CK, control group; HF, heart failure. Different lower letters above each boxplot showed the significant differences at *p* < 0.05.

**Figure 4:** Effects of cardiac contractility modulation (CCM) on mTOR, p-mTOR, GSK-3*β*, and TORC2 expression in different rabbit myocardial tissues under different treatments. (a) mTOR expression; (b) p-mTOR expression; (c) GSK-3*β* expression; (d) TORC2 expression; and (e) western blot images of mTOR, p-mTOR, GSK-3*β*, and TORC2. CK, control group; HF, heart failure. Different lower letters above each boxplot showed the significant differences at *p* < 0.05.

**Table 1:** Effects of cardiac contractility modulation (CCM) on the experimental rabbit body weight, heart weight, and heart rate (*n* = 27).

Group	Body weight (kg)	Heart weight (g)	Heart rate (bpm)
Control	3.2 ± 0.4^a†^	121 ± 14^a^	228 ± 6^a^
HF	2.5 ± 0.2^c^	86 ± 9^b^	258 ± 11^b^
CCM	2.9 ± 0.1^b^	111 ± 20^a^	240 ± 19^a^
ANOVA			
	Body weight	Heart weight	Heart rate
Treatment^‡^	0.021	0.001	0.011

Data are presented as mean ± SEM and analyzed by Mixed Proc with SAS software. HF; heart failure. ^†^Different letters in each column shows the significant differences at *p* < 0.05. ^‡^Treatment included control, heart failure, and cardiac contractility modulation groups.

## Data Availability

The original data used to support the findings of this study are available from the corresponding author upon request.
